The article "Efficacy and Safety of Shuganjieyu Capsule Alone or in Combination with Other Antidepressants in the Treatment of Postpartum Depression: A Meta-Analysis" was published in 2022. Journal: Evid Based Complement Alternat Med.

# Efficacy and Safety of Shuganjieyu Capsule Alone or in Combination with Other Antidepressants in the Treatment of Postpartum Depression: A Meta-Analysis

**DOI:** 10.1155/2022/5260235

**Published:** 2022-07-07

**Authors:** Lingning Wang, Yan Fan, Jiangmen He, Heng Liu, Feng Chen, Hongying Dan, Juan Zhao, Jiao Zhang, Tao Wang, Xinru Liu

**Affiliations:** ^1^Department of Obstetrics and Gynecology Clinics, West China Second University Hospital, Sichuan University, Chengdu 610041, China; ^2^Key Laboratory of Birth Defects and Related Diseases of Women and Children (Sichuan University), Ministry of Education, Chengdu 610041, China; ^3^Key Laboratory of Obstetric & Gynecologic and Pediatric Diseases of Sichuan Province, Chengdu 610041, China; ^4^Department of Pediatrics, West China Second University Hospital, Sichuan University, Chengdu 610041, China

## Abstract

**Objective:**

To evaluate the efficacy and safety of Shuganjieyu capsule alone or in combination with other antidepressants in the treatment of postpartum depression.

**Methods:**

Related control and randomized studies till August 1, 2021, were retrieved from the following databases: PubMed, Cochrane, CNKI, CMB, Wan-Fang, and VIP. Outcomes included HAMD reduction from baseline, response rate, and adverse events rate. Review Manager 5.3 was used in the present meta-analysis.

**Results:**

16 studies including 1409 participants were included in the present study. In comparison of single Shuganjieyu capsule versus regular antidepressant, 8, 6, and 4-week HAMD reduction of the Shuganjieyu group were significantly higher (8-week MD: 3.1 (1.54, 4.66), *p* < 0.0001; 6-week MD: 0.71 (0.10, 1.31), *p*=0.02; and 4-week MD: 0.82 (0.34, 1.30), *p*=0.0008), response rates were comparable for the two groups (OR: 1.51 (0.87, 2.63), *p*=0.014), and the adverse event rate of the Shuganjieyu group was significantly lower (OR: 0.22 (0.15, 0.32), *p* < 0.00001). In comparison of combination of Shuganjieyu capsule with regular antidepressant versus regular antidepressant alone, the 8, 6, 4, 2, and 1-week HAMD reduction and response rate of combination of Shuganjieyu with the regular antidepressant group were significantly larger (8-week MD: 3.2 (1.34, 5.06), *p*=0.0007; 6-week MD: 4.00 (2.72, 5.28), *p* < 0.00001; 4-week MD: 3.33 (1.94,4.73), *p* < 0.00001; 2-week MD: 2.69 (1.34, 4.03), *p* < 0.0001; 1-week MD: 2.27 (0.69, 3.86), *p*=0.005; and response rate OR: 4.69 (2.27, 9.68), *p* < 0.0001) and the adverse event rate was comparable for the two groups (OR: 1.26 (0.73, 2.17), *p*=0.41).

**Conclusion:**

Compared with regular antidepressants, single Shuganjieyu capsule has similar efficacy and better safety profile; when Shuganjieyu capsule is combined with regular antidepressants, the efficacy is improved significantly without increasing adverse events. Therefore, Shuganjieyu capsule was effective and safe for postpartum, making it worth further investigation and popularization.

The article "Efficacy and Safety of Shuganjieyu Capsule Alone or in Combination with Other Antidepressants in the Treatment of Postpartum Depression: A Meta-Analysis" was published in 2022. Journal: Evid Based Complement Alternat Med.

## 1. Introduction

Postpartum depression (PPD) is a common complication among mothers after childbirth. The prevalence rate of postpartum depression mainly ranged between 3.1% and 57.2% all over the world [1], and this rate was estimated to be 5.9%–26% in China [2–8]. Postpartum depression is associated with many serious adverse effects. It leads to poor quality of life of adult mother [9] and is a risk factor for postpartum suicide [10]. Furthermore, it also adversely affects long-term emotional [11], intellectual [12], and cognitive development of children [13, 14]. Current treatment strategies for PPD mainly include pharmacological interventions, psychological intervention, physiotherapy, and complementary therapies [15]. Determination of treatment strategy mainly depends on the category and severity of PPD. Efficacy and potential adverse effect among mothers and infants shall be comprehensively evaluated. Pharmaceutical therapies have included antidepressants, hormone, and Traditional Chinese Medicine (TCM).

Antidepressants remain important treatment options for PPD. Current antidepressants mainly included selective serotonin reuptake inhibitor drugs (SSRIs), tricyclic antidepressant (TCAs), and monoamine oxidase inhibitor (MAOI). SSRIs are first-line antidepressants. Due to few adverse effect, comparable efficacy with traditional antidepressants, and good tolerance, SSRIs are also often selected in PPD treatment. When using TCAs for PPD, plasma concentration and impact on breast milk shall be closely monitored; response rate and effective rate in PPD patients receiving SSRIs were higher than those receiving TCAs [16]. MAOIs are usually not used in PPD treatment due to relatively more adverse effect [17]. Except traditional antidepressants, brexanolone, a positive metamorphosis regulator of gamma-aminobutyric acid A receptor, showed to be effective in the treatment of moderate and severe PPD in recent study [18]. Estrogen is revealed to be associated with PPD, but its application in PPD treatment is not evidenced yet [19]. In China, many PPD patients would select TCM or acupuncture for treatment. A meta-analysis had included 15 Chinese herbal medicine (CHM) studies and 3 acupuncture studies and found that CHM alone or combined with antidepressants could relieve depression symptom; acupuncture was comparable with antidepressant, but with few adverse events [20].

Though antidepressants are first-line drug for PPD, antidepressants-associated side effects significantly affect the quality of life and compliance of mothers. Moreover, active components of most antidepressants can transfer into breast milk through passive diffusion, which may influence breastfed infants [21]. Though current studies showed that the application of antidepressants during breastfeeding was associated with very few obvious adverse events in infants [22,23], the sample sizes of these studies were small and evaluation duration was short, so the potential impact of antidepressants on infant through breastfeeding still could not be completely excluded. Therefore, among PPD patients who breastfed their infants, application of antidepressant shall be cautious, for example, selecting drugs with good safety profile, avoiding combination of two or more antidepressants, starting with low dosage, combination with other therapy to reduce dosage of antidepressant, and so on [24]. TCM has long history and accumulated abundant experience of PPD treatment, so its investigation might provide novel strategy or solution in this topic.

The article "Efficacy and Safety of Shuganjieyu Capsule Alone or in Combination with Other Antidepressants in the Treatment of Postpartum Depression: A Meta-Analysis" was published in 2022. Journal: Evid Based Complement Alternat Med.

Shuganjieyu capsule was a Chinese Patent Medicine (CPM) prepared from *Hypericum perforatum* L. and Radix Acanthopanacis Senticosi. It was the first CPM approved by State Food and Drug Administration (SFDA) for treatment of depression. In view of TCM, it has the function of “soothing liver and relieving depression, clearing away heat and dampness, detumescence and soothing breast” [25]. The antidepressant effect of *Hypericum perforatum* L. (St. John's wort) has also been recognized in many other countries and is widely used for treatment of depression [26]. According to the meta-analysis based on 29 trials including 5489 patients, *Hypericum perforatum* L. extracts have similarly efficacy but less side effects compared with standard antidepressants [26]. On the other hand, Radix Acanthopanacis Senticosi was recorded early in ancient pharmacological work “Supplementary Records of Famous Physicians” by Tao Hongjing in Han Dynasty [26]. In TCM opinion, it has the functions of “supplementing qi, strengthening spleen, tonifying kidney and calming nerves” [27] and is clinically used for treatment of depression, neurasthenia, and neurosis in China [28]. Pharmacological studies indicated that Radix Acanthopanacis Senticosi has effect of sedation, antifatigue, and promotion of cellular and humoral immunity [28]. Clinical studies showed that acanthopanax senticosus injection was effective in treatment of depression [29], has comparable efficacy but much less side effect compared with traditional antidepressants, including flupentixol and melitracen tablets and imipramine [30,31]. Prepared with *Hypericum perforatum* L. and Radix Acanthopanacis Senticosi, Shuganjieyu capsule is widely used in the treatment of depression in Chinese hospitals and its efficacy is evidenced for major depression, geriatric depression, and poststroke depression [32–38].

The article "Efficacy and Safety of Shuganjieyu Capsule Alone or in Combination with Other Antidepressants in the Treatment of Postpartum Depression: A Meta-Analysis" was published in 2022. Journal: Evid Based Complement Alternat Med.

There are a number of studies investigating Shuganjieyu capsule for PPD, but very few of them are published in English journals, so international researchers knew little about it. Therefore, we performed this meta-analysis to systematically review and evaluate the efficacy and safety of Shuganjieyu capsule in the treatment of PPD, which may also provide international researchers with a good access to knowing about Shuganjieyu capsule in PPD, thus potentially providing new treatment strategy and solution for PPD.

## 2. Materials and Methods

### 2.1. Inclusion and Exclusion Criteria

The inclusion criteria include the following: (1) type of study: randomized and control study; (2) type of participant: patients who developed depression within 6 weeks after delivery; meet the diagnosis criteria of depression defined by the Diagnostic and Statistical Manual of Mental Disorder IV (DSM-IV); regular physical examination result at inclusion was normal; did not use antidepressant and psychiatric drugs before; no alcohol or other substance addict; no serious suicidal tendency; provided informed consent; (3) type of intervention: patients in the control group received regular antidepressants; patients in the experimental group received Shuganjieyu capsule alone or combined with the antidepressant used in the control group; and (4) type of outcome measurement: at least one of HAMD reduction from baseline, response rate, and adverse events rate was evaluated.

The exclusion criteria include the following: (1) experimental drug Shuganjieyu was not in the form of capsule; (2) other drugs or treatment methods were used, such as acupuncture, massage, transcranial magnetic stimulation, and so on; and (3) retrospective study or single arm study was excluded.

### 2.2. Retrieval Strategy

We search the relative studies published till August 1, 2021, using the following databases: PubMed, Embase, and four Chinese medical databases: CNKI, CBM, Wan-Fang, and VIP. The retrieval terms included “postpartum depression,” “Shuganjieyu” or “Shugan Jieyu.” For the Chinese medical databases, corresponding Chinese counterparts for these terms were used. The potential references of retrieved articles were manually searched.

### 2.3. Literature Screening, Data Extraction, and Quality Assessment

Two authors screened the retrieved article, respectively, following a unified screening standard. Title, abstract, duplication, and main text of each retrieved article were examined. The screening results of the two authors were compared and the final inclusion was determined through discussion. When agreement cannot be reached, a third experienced author was invited to make final decision.

The article "Efficacy and Safety of Shuganjieyu Capsule Alone or in Combination with Other Antidepressants in the Treatment of Postpartum Depression: A Meta-Analysis" was published in 2022. Journal: Evid Based Complement Alternat Med.

The following information of each included article was collected: publication year, author name, number of participants, age of participants, treatment duration, baseline HAMD, intervention in the experimental group and control group, and outcome measurements.

Cochrane risk-of-bias tool was used for quality assessment. For each study, the random sequence generation, allocation concealment, blinding of participants and personnel, blinding of outcome assessment, incomplete outcome data, and selective reporting were assessed and graded as low risk, unclear risk, and high risk.

### 2.4. Outcome Measurements

The depression symptoms were assessed using Hamilton Depression Scale-17 items (HAMD-17). 8-week/6-week/4-week/2-week/1-week HAMD reduction from baseline = HAMD score at baseline-HAMD score at 8 weeks/6 weeks/4 weeks/2 weeks/1 week. Response rate = number of patients who responded to treatment showing HAMD reduction no less than 50%/total number of patients. Adverse events rate = number of adverse events/total number of patients.

### 2.5. Statistical Analysis

RevMan5.3 was used to perform the present meta-analysis. Odd ratio (OR) for response rate and adverse events rate and mean difference (MD) for HAMD reduction from baseline were calculated and compared between the experimental group and control group. *p* < 0.05 was considered statistically significant. Heterogeneity test was made to analyze the difference between included studies. If the heterogeneity was not significant (*p* > 0.1, *I*^2^ < 50%), fixed effect model was used; if the heterogeneity was significant (*p* < 0.1, *I*^2^ > 50%), the random effect model was applied. Subgroup analysis was made according to the regular antidepressants. Publication bias was estimated with funnel plot.

## 3. Results

### 3.1. Literature Screening Results and Characteristics of Included Studies

Following the retrieval strategy described above, 27 articles were retrieved, among which, 18 can be retrieved from CNKI, 15 can be retrieved from Wan-Fang, 8 can be retrieved from VIP, 10 can be retrieved from CBM, and 0 from PubMed, EMBASE, and Cochrane Library. After duplicate checking, 1 article was excluded. After title and abstract examination, 4 articles were excluded. After main-text examination, 6 articles were excluded for the following reasons: acupuncture treatment was combined in 1 article; Shuganjieyu soup rather than capsule was used in 2 articles; transcranial magnetic stimulation was used in 1 article; and none of 17-item-HAMD reduction, response rate, and adverse events rate was evaluated in 2 articles. Finally, 16 articles were included in our meta-analysis. The PRISMA 2009 flowchart of the selection process is shown in Figure 1.

The article "Efficacy and Safety of Shuganjieyu Capsule Alone or in Combination with Other Antidepressants in the Treatment of Postpartum Depression: A Meta-Analysis" was published in 2022. Journal: Evid Based Complement Alternat Med.

The characteristics of included studies are given in Table 1. Among the 16 studies [39–54], 10 studies compared single Shuganjieyu capsule and one regular antidepressant [39–48]; 6 studies compared combination of Shuganjieyu capsule and regular antidepressant versus regular antidepressant alone [49–54]. The regular antidepressant included citalopram, paroxetine, fluoxetine, and sertraline. Shuganjieyu capsules was administered as follows in 9 studies [39–45, 50, 51]: initial 0.36–0.72 g/d, increased to 1.08–1.44 g/d in following 1–2 weeks. In the remaining 7 studies, Shuganjieyu was administered as follows: 1.44 g/d [46–49, 52–54]. The dosage of citalopram ranged between 20 and 40 mg/d [39–45, 49–51] and could be adjusted to no more than 60 mg/d [47]; the dosage of paroxetine ranged from 10 mg/d to 50 mg/d [48, 53, 54]; the dosage of fluoxetine was 20 mg/d [46]; the dosage of sertraline was 50 mg/d and could be adjusted to no more than 100 mg [52]. The treatment length arranged from 6 weeks to 8 weeks. The HAMD-17 was used to assess depression severity in 14 studies, except one study used different scale for depression assessment [43] and one study assessed anxiety symptom rather than depression symptom [50].

### 3.2. Quality Assessment Results of Included Studies

The quality assessment results are shown in Figures 2 and 3. 5 studies using random number table [40,47,48,51,53] were rated as low risk, 2 studies using odd or even number to generate random sequence [45,49], and 3 studies making allocation on intervention [41,50,52] were rated as high risk, and the remaining studies that reported randomization but did not describe the specific method of random sequence generation were rated as unclear. Details on blindness of allocation, participants and personnel, and outcome assessment were not described by all the 16 studies, so the blindness of allocation and assessment were all rated as unclear, and the blindness of participants and personnel were rated as high risk considering the general practice in hospital of China. Among the 16 studies, 2 study reported rate of dropout or loss to follow up [36,42]; other 14 studies reported all patients had completed the trial; 4 studies included in analysis for adverse event rate did not report the rate of each adverse event [39,42,45,47]; however, these studies aimed to evaluate the score of Treatment Emergent Symptom Scale (TESS) rather than adverse events rates, so they were rated as unclear for bias of incomplete data report. The selective reporting and other risk of bias were rated as unclear for all 16 studies.

The article "Efficacy and Safety of Shuganjieyu Capsule Alone or in Combination with Other Antidepressants in the Treatment of Postpartum Depression: A Meta-Analysis" was published in 2022. Journal: Evid Based Complement Alternat Med.

## 4. Outcomes

### 4.1. Comparison of Single Shuganjieyu Capsule versus Regular Antidepressants

#### 4.1.1. HAMD Reduction from Baseline

In total, 6 studies compared 6-week HAMD reduction in the Shuganjieyu group and regular antidepressant group (Figure 4). 5 studies compared Shuganjieyu citalopram, with 197 patients in the Shuganjieyu group and 193 patients in the citalopram group. The heterogeneity between the studies was not significant (*p* = 0.93, *I*^2^ = 0%). The difference of HADM reduction between the two groups was not significant (*p* = 0.05). 1 study compared Shuganjieyu and fluoxetine. The HAMD reduction of Shuganjieyu was not significantly different from that of the fluoxetine group (*p* = 0.21). The meta-analysis for the 6 studies was performed. The heterogeneity between the studies was not significant (*p* = 0.95, *I*^2^ = 0%). The test for the overall effect showed that the HAMD reduction of the Shuganjieyu group was significantly larger than that in the regular antidepressant group (*p* = 0.02). The difference between the subgroups was not significant (*p* = 0.60, *I*^2^ = 0%).

Comparison of 8, 4, 2, 1-week HAMD reduction among patients receiving Shuganjieyu capsule versus regular antidepressant was also made (Table 2). Analysis for 8-weekHAMD reduction included 1 study, with 77 patients. 8-week HAMD reduction was significantly larger in the Shuganjieyu group (*p* < 0.0001). Analysis for 4-week HAMD reduction included 7 studies, with 563 patients. The heterogeneity between studies was significant (*p* = 0.04, *I*^2^ = 55%). The test for he overall effect indicated 4-week HAMD reduction of the Shuganjieyu capsule group was significantly higher than that of the regular antidepressant group (*p* = 0.0008). Analysis for 2-week HAMD reduction included 6 studies, with 486 patients. The heterogeneity was not significant (*p* = 0.22, *I*^2^ = 29%). The test for he overall effect indicated that 2-week HAMD reduction of the Shuganjieyu group was not significantly different from that of regular antidepressant (*p* = 0.27). Analysis for 1-week HAMD reduction included 5 studies, with 390 patients. The heterogeneity was significant (*p* = 0.08, *I*^2^ = 71%). The test for overall effect indicated that 1-week HAMD reduction of the Shuganjieyu group was not significantly different from that of the regular antidepressant group (*p* = 0.35). In the sensitivity test for the analysis of 1-week HAMD reduction, when the study by Zhang Xiaoqin was removed, the heterogeneity between studies was not significant anymore (*p* = 0.45, *I*^2^ = 0%).

The article "Efficacy and Safety of Shuganjieyu Capsule Alone or in Combination with Other Antidepressants in the Treatment of Postpartum Depression: A Meta-Analysis" was published in 2022. Journal: Evid Based Complement Alternat Med.

#### 4.1.2. Response Rate

In total, 6 studies compared response rate among PPD patients receiving Shuganjieyu capsules versus regular antidepressants, which include paroxetine, citalopram, fluoxetine (Figure 5).

1 study compared Shuganjieyu capsule and paroxetine, which included 39 patients in the Shuganjieyu capsule group and 38 patients in the paroxetine group. The response rate of the Shuganjieyu group was significantly higher (*p* = 0.02). 1 study compared Shuganjieyu capsule and fluoxetine, which included 48 patients in the Shuganjieyu capsule group and 48 patients in the fluoxetine group. The response rate of the Shuganjieyu group was not significantly different from that of fluoxetine (*p* = 0.75). 4 studies compared Shuganjieyu and citalopram, which included 164 patients in the Shuganjieyu group and 160 patients in the citalopram group. The heterogeneity analysis indicated that there was no significant heterogeneity between the included studies (*p* = 0.93; *I*^2^ = 0%). The meta-analysis result indicated that response rate in the Shuganjieyu group is not significantly different with that in the citalopram group (*p* = 0.54).

The meta-analysis for the 6 studies was also performed. The heterogeneity analysis indicated the heterogeneity between the 6 studies was not significant (*p* = 0.49; I^2^ = 0%). The test for overall effect indicated that response rate of the Shuganjieyu group is not significantly different with that of regular antidepressant group (*p* = 0.14). The difference between the subgroup is not significant (*p* = 0.14, *I*^2^ = 49.8%). Funnel plot was adopted to estimate the publication bias, and the result suggested no obvious publication bias (Figure 6).

#### 4.1.3. Adverse Events Rates

In total, 10 studies compared overall adverse events rate in patients receiving Shuganjieyu and regular antidepressant (Figure 7). 8 studies compared Shuganjieyu and citalopram, with 360 patients in the Shuganjieyu group and 356 patients in citalopram group. The heterogeneity between the 8 studies was not significant (*p* = 0.48, *I*^2^ = 0%). The test for overall effect indicated that the AE rate of the Shuganjieyu group was significantly lower than that of citalopram group (*p* < 0.00001). 1 study compared Shuganjieyu and paroxetine. The AE rate of the Shuganjieyu group was significantly lower than that of the paroxetine group (*p* = 0.002). 1 study compared Shuganjieyu and fluoxetine. The AE rate of the Shuganjieyu group was significantly lower than that of the fluoxetine group (*p* = 0.03). The meta-analysis with all the 10 studies was also performed. The heterogeneity between the studies was not significant (*p* = 0.49, *I*^2^ = 0%). The test for he overall effect indicated that the AE rate of the Shuganjieyu group was significantly lower (*p* < 0.00001). The difference between the subgroups was not significant (*p* = 0.42, *I*^2^ = 0%).

The article "Efficacy and Safety of Shuganjieyu Capsule Alone or in Combination with Other Antidepressants in the Treatment of Postpartum Depression: A Meta-Analysis" was published in 2022. Journal: Evid Based Complement Alternat Med.

Summary and comparison of each adverse event are given in Table 3. The comparison of adverse event rate among patients receiving Shuganjieyu versus citalopram included 4 studies, with 210 participants in the experimental group and 210 participants in the control group (Table 3). The rates of dizziness, insomnia, nausea/vomiting, and tachycardia were significantly lower in the Shuganjieyu group compared with that in the citalopram group (all *p* < 0.05). The rates of dry mouth, constipation, hand tremor, anorexia, and agitation were similar for the Shuganjieyu group and citalopram group (all *p* > 0.05).

The comparison of each adverse event among the patients receiving Shuganjieyu versus paroxetine included 1 study, with 39 patients in the Shuganjieyu group and 38 patients in the paroxetine group (Table 3). The rate of dry mouth was significantly lower in the Shuganjieyu group compared with paroxetine (*p* = 0.019). The rates of dizziness, insomnia, and nausea/vomiting were similar for two groups (all *p* > 0.05).

The comparison of each adverse event among the patients receiving Shuganjieyu versus fluoxetine included 1 study, with 48 patients in the Shuganjieyu group and 48 patients in the fluoxetine group (Table 3). The rate of insomnia was significantly lower in the Shuganjieyu group (*p* = 0.014). The rates of dizziness, nausea/vomiting, somnolence, and anorexia were similar for the two groups (all *p* > 0.05).

### 4.2. Comparison of Shuganjieyu Capsule plus Regular Antidepressants versus Regular Antidepressants

#### 4.2.1. HAMD Reduction from Baseline

In total, 3 studies compared 6-week HAMD reduction in patients receiving Shuganjieyu plus regular antidepressant versus regular antidepressant alone (Figure 8). 2 studies compared Shuganjieyu and citalopram, with 88 patients in the Shuganjieyu plus citalopram group and 88 patients in the citalopram group. The heterogeneity was not significant (*p* = 0.16, *I*^2^ = 48%). The test for overall effect indicated that the 6-week HAMD reduction of the Shuganjieyu plus citalopram group was significantly larger than that of the citalopram group (*p* < 0.00001). 1 study compared Shuganjieyu plus paroxetine and paroxetine. 6-week HAMD reduction was significantly higher in the Shuganjieyu plus paroxetine group compared with the paroxetine alone group (*p* = 0.02). Meta-analysis was performed with all the 3 studies. The heterogeneity was not significant (*p* = 0.38, *I*^2^ = 0%). The test for the overall effect indicated that the 6-week HAMD reduction of Shuganjieyu plus regular antidepressant was significantly higher than that of the regular antidepressant alone group (*p* < 0.00001). The difference between subgroups was not significant (*p* = 0.92, *I*^2^ = 0%).

The article "Efficacy and Safety of Shuganjieyu Capsule Alone or in Combination with Other Antidepressants in the Treatment of Postpartum Depression: A Meta-Analysis" was published in 2022. Journal: Evid Based Complement Alternat Med.

Comparison of 8, 4, 2, and 1-week HAMD reduction among the patients receiving Shuganjieyu plus regular antidepressant versus regular antidepressant alone was also performed (Table 4). The analysis for 8-weekHAMD reduction included 1 study. The 8-week HAMD reduction was significantly larger in the Shuganjieyu plus paroxetine group compared with paroxetine alone group (*p* = 0.0007). The analysis for 4-week HAMD reduction included 2 studies, with 156 participants. The heterogeneity between studies was not significant (*p* = 0.4, *I*^2^ = 0%). The test for overall effect indicated 4 weeks HAMD reduction of the Shuganjieyu plus regular antidepressant combination group was significantly larger than that of the antidepressant alone group (*p* < 0.00001). The analysis for 2-week HAMD reduction included 2 studies, with 156 participants. The heterogeneity between the studies was not significant (*p* = 0.31, *I*^2^ = 4%). The test for the overall effect indicated 2-weekHAMD reduction of the Shuganjieyu plus regular antidepressant combination group was significantly larger than that of the antidepressant alone group (*p* < 0.0001). The analysis for 1-week HAMD reduction included 2 studies, with 116 patients. The heterogeneity between studies was not significant (*p* = 0.66, *I*^2^ = 0%). The test for the overall effect indicated that 1-week HAMD reduction of the Shuganjieyu plus antidepressant combination group was significantly larger than that of the antidepressant alone group (*p* = 0.005).

#### 4.2.2. Response Rate

In total, 5 studies had compared the response rate among the patients receiving regular antidepressant + Shuganjieyu or regular antidepressant alone (Figure 9). The regular antidepressants included paroxetine, citalopram, and sertraline.

2 studies compared Shuganjieyu plus paroxetine versus paroxetine alone, with 80 patients in each group (Figure 9). The heterogeneity between the 2 studies was not significant (*p* = 0.37, *I*^2^ = 0%). Test for overall effect indicated that the response rate of the Shuganjieyu plus regular antidepressant group was significantly higher than that of the regular antidepressant alone group (OR = 3.92 (1.57, 9.78); *p* = 0.03). 2 studies compared Shuganjieyu plus citalopram versus citalopram alone, with 88 patients in each group. The heterogeneity between the studies was not significant (*p* = 0.63, *I*^2^ = 0%). The test for the overall effect indicated that the response rate of the Shuganjieyu plus regular antidepressant group was significantly higher than that of the regular antidepressant alone group (OR = 4.90 (1.3, 18.54); *p* = 0.02). 1 study compared Shuganjieyu plus sertraline versus sertraline alone, with 32 patients in each group. The response rate of the Shuganjieyu plus sertraline group was not significantly higher than that of the sertraline alone group (*p* = 0.09).

The article "Efficacy and Safety of Shuganjieyu Capsule Alone or in Combination with Other Antidepressants in the Treatment of Postpartum Depression: A Meta-Analysis" was published in 2022. Journal: Evid Based Complement Alternat Med.

The meta-analysis for the 5 studies was performed (Figure 9). The heterogeneity between the studies was not significant (*p* = 0.79, *I*^2^ = 0%). THe test for the overall effect indicated that the response rate of the Shuganjieyu plus regular antidepressant group was significantly higher than that of the regular antidepressant group (OR = 4.69 (2.27, 9.68); *p* < 0.0001). The difference between the subgroups was not significant (*p* = 0.74, *I*^2^ = 0%). Funnel plot did not exhibit obvious publication bias (Figure 10).

#### 4.2.3. Adverse Events Rates

In total, 4 studies compared AE rate among patients receiving Shuganjieyu plus regular antidepressant or regular antidepressant alone (Figure 11). 3 studies compared Shuganjieyu plus citalopram and citalopram, with 148 patients in the Shuganjieyu plus citalopram group and 148 patients in the citalopram alone group. The heterogeneity was not significant (*p* = 0.76, *I*^2^ = 0%). The AE rate in the Shuganjieyu plus citalopram group was not significantly different from that in the citalopram alone group (*p* = 0.53). 1 study compared Shuganjieyu plus sertraline and sertraline alone. The AE rate in the Shuganjieyu plus sertraline group was not significantly different from that in the sertraline alone group (*p* = 0.55). The meta-analysis for the 4 studies was also performed, with 180 patients in the Shuganjieyu plus regular antidepressant group and 180 patients in the regular antidepressant alone group. The heterogeneity between the studies was not significant (*p* = 0.9, *I*^2^ = 0%). The AE rate in the Shuganjieyu plus regular antidepressant group was not significantly different from that in the regular antidepressant alone group (*p* = 0.41). The difference between subgroups was not significant (*p* = 0.80, *I*^2^ = 0%).

The summary and comparison of each adverse event are given in Table 5. The comparison of Shuganjieyu plus citalopram versus citalopram included 3 studies, with 148 patients in the Shuganjieyu plus citalopram group and 148 patients in the citalopram group. The rates of dry mouth, headache, dizziness, nausea/vomiting, blurred vision, somnolence, and fatigue were similar for the two groups (all *p* > 0.05). The comparison of Shuganjieyu plus sertraline and sertraline included 32 patients in the Shuganjieyu plus sertraline group and 32 patients in the sertraline group. The rates of flatulence, nausea/vomiting, and somnolence were not significantly different for the two groups (all *p* > 0.05).

The article "Efficacy and Safety of Shuganjieyu Capsule Alone or in Combination with Other Antidepressants in the Treatment of Postpartum Depression: A Meta-Analysis" was published in 2022. Journal: Evid Based Complement Alternat Med.

## 5. Discussion

Several clinical studies had investigated Shuganjieyu capsule for the treatment of postpartum depression. In this meta-analysis, we evaluated efficacy and safety of Shuganjieyu capsule used alone or in combination with regular antidepressant in treatment of PPD.

The result of the present analysis demonstrated in comparison of single Shuganjieyu capsule versus regular antidepressant, 8-, 6-, and 4-week HAMD reduction of the Shuganjieyu group were significantly higher, response rates were comparable for the two groups, and the adverse event rate of the Shuganjieyu group was significantly lower. In comparison of combination of Shuganjieyu capsule with regular antidepressant versus regular antidepressant alone, the 8, 6, 4, 2, 1-week HAMD reduction and response rate of combination of Shuganjieyu with the regular antidepressant group were significantly larger and the adverse event rate were comparable for the two groups. These results demonstrated that, compared with regular antidepressants, Shuganjieyu capsule has similar efficacy and significantly better safety profile; when Shuganjieyu capsule is combined with regular antidepressants, the efficacy could be improved significantly without increasing adverse events.

According to the result of analysis for HAMD reduction among patients receiving Shuganjieyu capsule alone versus regular antidepressant (Table 2), the 1 and 2-week HAMD reduction of the Shuganjieyu group were slightly higher than those of the regular antidepressant group but showed no significance, which indicated that onset of action of Shuganjieyu was similar to citalopram or fluoxetine. Previous study revealed that early onset of action was associated with higher remission rate in the treatment of depression [55]. Therefore, Shuganjieyu capsule might be similar to citalopram or fluoxetine in aspect of rapid onset.

The heterogeneity between studies in most comparisons was not significant, except in the analysis of 4-week (*p* = 0.04, *I*^2^ = 55%) and 1-week (*p* = 0.08, *I*^2^ = 71%) HAMD reduction among patients receiving single Shuganjieyu capsule versus regular antidepressants. The subgroup analysis result of 4-week HAMD reduction (subgroup difference: *p* = 0.02, *I*^2^ = 73.9%) indicated the regular antidepressant compared was a source of the heterogeneity. The heterogeneity may result from the different antidepressant effect of different kinds of antidepressants. In the analysis of 1-week HAMD reduction, there is only one type of regular antidepressant of citalopram, so sensitivity test was performed, which indicated that when the study by Zhang Xiaoqin et al. was removed, the heterogeneity was not significant anymore (*p* = 0.45, *I*^2^ = 0%). The dosage of Shuganjieyu capsule was 1.44 g/d in the study by Zhang Xiaoqin, and the dosage in other included studies was initially 0.36 g–0.72 g/d and increased to 1.08–1.44 g/d in 1–2 weeks, so we speculate the initial higher dosage of Shuganjieyu in the study by Zhang Xiaoqin contributed to the heterogeneity in the analysis of 1-week HAMD reduction.

The article "Efficacy and Safety of Shuganjieyu Capsule Alone or in Combination with Other Antidepressants in the Treatment of Postpartum Depression: A Meta-Analysis" was published in 2022. Journal: Evid Based Complement Alternat Med.

Our analysis had demonstrated that Shuganjieyu capsule showed a good safety profile. The adverse events related to Shuganjieyu capsule mainly include dry mouth, dizziness, insomnia, constipation, nausea/vomiting, and anorexia (Table 3), but most of the ADRs were lower than those in the regular antidepressants group. Previous studies supported this conclusion. According to the meta-analysis evaluating Shuganjieyu capsule for major depression disorder in 595 adult participants, Shuganjieyu capsule alone is superior to placebo in terms of from baseline of traditional Chinese medicine syndrome scale score, and Shuganjieyu plus venlafaxine is also superior to venlafaxine alone in terms of safety [35]. Furthermore, in another meta-analysis evaluating Shuganjieyu capsule for the treatment of mild or moderate depression that included 990 patients, adverse events rats of the Shuganjieyu group were significantly lower than that of the group of regular antidepressants that included mirtazapine, venlafaxine, flupentixol and melitracen, sertraline, paroxetine, fluoxetine, and citalopram [56]. Consistent conclusions regarding safety of Shuganjieyu capsule had also been achieved by other meta-analyses [57,58]. These results suggested Shuganjieyu capsule was very safe and suitable for patients with more safety concerns, such as those with PPD or chronic disease.

A number of studies had explored the mechanism of Shuganjieyu capsules for treatment of postpartum depression. *Hypericum perforatum* L. has been known for its antidepression effect and received much attention by researchers. It may increase concentration of 5-hydroxytryptamine (5-HT), norepinephrine (NA), dopamine (DA), and glutamic acid [59,60], inhibiting gamma-aminobutyric acid (GABA) and *N*-methyl-D-aspartic acid (NMDA) receptors [61] in treatment of depression. Acanthopanacis Senticosi has shown its antidepression effect in some clinical studies [62,63]. It may have protection effect for dopamine neurons and [64]; increase hippocampus BDNF expression level and improve study memory function of depression model rats [65]; and increase tyrosine hydroxylase (TH) and tyrosine hydroxylase (TPH) expression level in hippocamp of depressed rats [66]. The laboratory investigation showed that Shuganjieyu capsule could regulate the function of DA, 5-HT, Glu, and GABA neurotransmitter system in medial prefrontal cortex (mPFC) and hippocampus area of rat model of depression [67]; could regulate expression level of transient receptor potential channel 6 (TRPC6), phosphorylated-cAMP response element binding protein (p-CREB) and brain-derived neurotrophic factor (BDNF) in frontal region and hippocampus area of rat model of depression [68–70]; and promoted recovery/regeneration of impaired neurons in hippocampus area of rat model of depression through downregulation of caspase-3 protein level [71,72]. Moreover, network pharmacology study showed Shuganjieyu capsule may affect 552 targets as well as MAPK pathway, TNF pathway, PI3K-Akt pathways, and so on in treatment of depression [73]. These results suggested that Shuganjieyu capsule may exert antidepression effect through multiple links and targets, having different mechanism from regular antidepressants.

The article "Efficacy and Safety of Shuganjieyu Capsule Alone or in Combination with Other Antidepressants in the Treatment of Postpartum Depression: A Meta-Analysis" was published in 2022. Journal: Evid Based Complement Alternat Med.

Currently, in PPD treatment in China, nonpharmaceutical therapy of psychological treatment and physical treatment are preferred; when pharmaceutical treatment was used, it is often combined with psychological treatment, or a combination of Western medicine and traditional Chinese medicine was adopted [74]. It is because usage of antidepressants needs to be cautious among PPD patients to avoid potential impact of antidepressants on mothers and infants. Except our founding of Shuganjieyu capsule in PPD, there are also a number of studies and meta-analyses confirmed efficacy and safety of Shuganjieyu capsules in treatment of mild or moderate depression [37], depression in old age [31], depression at acute stage [38], poststroke depression [32], and so on in single usage or in combination. These founding together with Shuganjieyu capsule had nature origin, making Shuganjieyu capsule a good alternative or complementary drug for regular antidepressant. However, current relative studies are not of high quality. Studies with more rigid design are needed to further confirm the effect of Shuganjieyu capsules.

This is the first meta-analysis evaluating efficacy and safety of Shuganjieyu capsule in the treatment of PPD. It may provide international researchers with a good access to the related studies carried out and mainly published in Chinese medical journals, thus assisting in development of potential new treatment strategy for PPD and target of future investigations. However, there are some limitations: (1) The quality of included studies was relatively poor. All studies did not provide details of blindness. These may lead to risk of bias. (2) All studies were performed in China and published in Chinese journals, which may result in certain bias. (3) Sample size: though 16 studies were included in the present meta-analysis, except the subgroup of citalopram, the sample size of subgroup analysis with fluoxetine, paroxetine, and sertraline is not large, which made it difficult to better analyze subgroups.

The article "Efficacy and Safety of Shuganjieyu Capsule Alone or in Combination with Other Antidepressants in the Treatment of Postpartum Depression: A Meta-Analysis" was published in 2022. Journal: Evid Based Complement Alternat Med.

## 6. Conclusion

The potential side effects of regular antidepressants in mothers and infants make it necessary to be cautious to determine pharmaceutical treatment. Our study indicated that Shuganjieyu capsule alone had similar efficacy and better safety profile compared with regular antidepressants; Shuganjieyu capsule combined with regular antidepressant had better efficacy compared with regular antidepressant, without significant increase of adverse effect. Considering its natural origin, Shuganjieyu capsule shall be a good option no matter for single usage or combination in treatment of PPD patients, which makes it worth further investigation and popularization.

## Figures and Tables

**Figure 1:** PRISMA 2009 flowchart of the selection process.

**Figure 2:** Risk of bias graph of included studies.

**Figure 3:** Summary of risk of bias of included studies.

**Figure 4:** Forest plot of 6 weeks HAMD reduction from baseline in PPD patients receiving Shuganjieyu capsule alone versus regular antidepressant.

**Figure 5:** Forest plot of response rate in patients receiving Shuganjieyu capsule alone versus regular antidepressant.

**Figure 6:** Funnel plot of response rate for the publication bias. Note: comparison = Shuganjieyu capsule versus regular antidepressants; outcome = response rate; antidepressants = citalopram, paroxetine, or fluoxetine.

**Figure 7:** Forest plot of adverse event rate in patients receiving Shuganjieyu capsule alone versus regular antidepressant.

**Figure 8:** Forest plot of 6-week HAMD reduction among the patients receiving combination of Shuganjieyu and regular antidepressant versus regular antidepressant.

**Figure 9:** Forest plot of response rate in patients receiving combination of Shuganjieyu capsule and regular antidepressant versus regular antidepressant.

**Figure 10:** Funnel plot of response rate for the publication bias. Note: comparison = Shuganjieyu capsule plus regular antidepressants versus regular antidepressants; outcome = response rate; antidepressants = citalopram, paroxetine, or sertraline.

The article "Efficacy and Safety of Shuganjieyu Capsule Alone or in Combination with Other Antidepressants in the Treatment of Postpartum Depression: A Meta-Analysis" was published in 2022. Journal: Evid Based Complement Alternat Med.

**Figure 11:** Forest plot of adverse events rate in patients receiving combination of Shuganjieyu capsule and regular antidepressant versus regular antidepressant.

**Table 1:** Characteristics of included studies.

First author	No.			Baseline HAMD	Treatment duration	Intervention		Measurements
	Year	*E*/*C*	Age			*C*	*E*	
Chen Zhibin [39]	2012	33/33	27 ± 5.6/26 ± 6.1	22.7 ± 2.8/22.6 ± 2.7	6 weeks	Citalopram 20–40 mg/d	SC 3–4 capsules/d	HAMD, ADR
Luo Yongjun [40]	2016	40/40	26.8 ± 4.1/27.3 ± 4.2	30.2 ± 6.5/28.9 ± 6.4	6 weeks	Citalopram 20–40 mg/d	SC 3–4 capsules/d	RR, HAMD, ADR
Qi Jipeng [41]	2019	40/40	27.51 ± 5.37/27.92 ± 5.03	22.7 ± 2.7/22.8 ± 2.6	6 weeks	Citalopram 20–40 mg/d	SC 3–4 capsules/d	RR, HAMD, ADR
Sun Linna [42]	2013	36/32	27.4 ± 5.3 (23–35)	22.8 ± 3.1/22.7 ± 2.9	6 weeks	Citalopram 20–40 mg/d	SC 3–4 capsules/d	HAMD, RR, ADR
Wang Shuai [43]	2020	100/100	28.12 ± 1.32/28.55 ± 1.58	15.69 ± 1.54/15.58 ± 1.54^*∗*^	6 weeks	Citalopram 20–40 mg/d	SC 3–4 capsules/d	ADR
Xia Jinhua [44]	2013	30/30	26.1 ± 6.2/27.4 ± 5.5	22.7 ± 2.8/22.6 ± 2.7	6 weeks	Citalopram 20–40 mg/d	SC 3–4 capsules/d	HAMD, ADR
Ye Qinghong [45]	2012	33/33	27 ± 5.6/26 ± 6.1	22.7 ± 2.8/22.6 ± 2.7	6 weeks	Citalopram 20–40 mg/d	SC 3–4 capsules/d	HAMD, ADR
Zhang Baojian [46]	2014	48/48	27.03 ± 5.12/26.72 ± 4.67	21.32 ± 4.34/20.65 ± 4.29	6 weeks	Fluoxetine 20 mg/d	SC 4 capsules/d	RR, ADR, HAMD
Zhang Xiaoqin [47]	2015	48/48	26.8 ± 4.3/25.9 ± 4.8	23.1 ± 2.6/22.9 ± 2.7	6 weeks	Citalopram 20–60 mg/d	SC 4 capsules/d	HAMD, RR, ADR
Qian Shuangfeng [48]	2014	39/38	25.7 ± 4.5/25.3 ± 4.4	21.2 ± 3.9/21.8 ± 4.1	8 weeks	Paroxetine 20 mg/d	SC 4 capsules/d	HAMD, RR, ADR
Hao Ruijun [49]	2015	28/28	27 ± 9/23.4 ± 3.2	24 ± 4/23 ± 4	6 weeks	Citalopram 20 mg/d	SC 4 capsules/d + treatment of C	HAMD, RR, ADR.
Liang Dongxu [50]	2020	60/60	29.65 ± 6.21/29.81 ± 6.54	Not provided	6 weeks	Citalopram 18–40 mg/d	SC 3–4 capsules/d + treatment of C	ADR
Qiu Lan [51]	2017	60/60	31.02 ± 10.11/32.26 ± 10.28	24.34 ± 6.78/24.91 ± 7.02	6 weeks	Citalopram 20–40 mg/d	SC 3–4 capsules/d + treatment of C	RR, HAMD, ADR
Jing Kaige [52]	2016	32/32	29.6 (26–37)	Not provided	8 weeks	Sertraline 50–150 mg/d	SC 4 capsules/d + treatment of C	RR, ADR
Chen Lizhen [53]	2019	30/30	26.89 ± 3.49/27.54 ± 3.28	23.59 ± 5.61/23.37 ± 5.52	6 weeks	Paroxetine 20–50 mg/d	SC 4 capsules/d + treatment of C	HAMD, RR
Jin Xiaoduo [54]	2013	50/50	26 ± 3/27 ± 2.5	23.9 ± 5.4/23.7 ± 5.5	8 weeks	Paroxetine 10 mg/d	SC 4 capsules/d + treatment of C	RR, HAMD

ADR, adverse drug reaction; HAMD, Hamilton Depression Scale; *E*, experimental group; *C*, control group; No., number; RR, response rate; SC, Shuganjieyu capsule; treatment of *C*, treatment of the control group. ^*∗*^Different depression scale.

The article "Efficacy and Safety of Shuganjieyu Capsule Alone or in Combination with Other Antidepressants in the Treatment of Postpartum Depression: A Meta-Analysis" was published in 2022. Journal: Evid Based Complement Alternat Med.

**Table 2:** Summary of comparisons of 1, 2, 4, and 6-week HAMD reduction among the patients receiving Shuganjieyu capsule versus regular antidepressants.

Outcome or subgroup	Studies	No. of patients	Heterogeneity (*p*/*I*^2^)	Subgroup difference (*p*/*I*^2^)	Mean difference	*P*
8-week HAMD reduction	1	77	Not applicable	Not applicable	3.10 (1.54, 4.66)	<0.0001
Vs. paroxetine	1	77	Not applicable	—	3.10 (1.54, 4.66)	<0.0001
6-week HAMD reduction	6	486	0.95/0%	0.60/0%	0.71 (0.10, 1.31)	0.02
Vs. citalopram	5	390	0.9/0%	—	0.65 (0.01,1.29)	0.05
Vs. fluoxetine	1	96	Not applicable	—	1.17 (−0.67, 3.01)	0.21
4-week HAMD reduction	7	563	0.04/55%	0.02/73.9%	0.82 (0.34, 1.30)	0.0008
Vs. citalopram	5	390	0.24/28%	—	0.51 (−0.03, 1.04)	0.06
Vs. paroxetine	1	77	Not applicable	—	2.60 (1.00, 4.20)	0.001
Vs. fluoxetine	1	96	Not applicable	—	1.82 (0.26, 3.38)	0.02
2-week HAMD reduction	6	486	0.22/29%	0.60/0%	0.24 (−0.19, 0.66)	0.27
Vs. citalopram	5	390	0.15/41%	—	0.21 (−0.23, 0.65)	0.35
Vs. fluoxetine	1	96	Not applicable	—	0.67 (−0.98, 2.32)	0.43
1-week HAMD reduction	5	390	0.08/71%	Not applicable	0.18 (−0.20, 0.56)	0.35
Vs. citalopram	5	390	0.08/71%	—	0.18 (−0.20, 0.56)	0.35

**Table 3:** Summary and comparison of each adverse event among the patients receiving Shuganjieyu capsule versus regular antidepressants.

Intervention	Shuganjieyu vs. citalopram in 4 studies^*∗*^ [36–38, 40]			Shuganjieyu vs. paroxetine in 1 study [44]			Shuganjieyu vs. fluoxetine in 1 study [42]		
Study	Experiment (*n* = 210)	Control (*n* = 210)	*P*	Experiment (*n* = 39)	Control (*n* = 38)	*P*	Experiment (*n* = 48)	Control (*n* = 48)	*P*
Flatulence	0	0	—	0	0	—	0	0	—
Dry mouth	2	3	0.653	0	5	0.019	0	0	—
Headache	0	0	—	0	0	—	0	0	—
Dizziness	2	8	0.055	1	4	0.156	1	1	1
Insomnia	5	18	0.005	0	2	0.147	1	8	0.014
Constipation	2	2	1.000	0	0	—	0	0	—
Hand tremor	1	0	0.317	0	0	—	0	0	—
Nausea/vomiting	5	25	0.000	1	4	0.156	2	3	0.646
Blurred vision	0	0	—	0	0	—	0	0	—
Tachycardia	1	14	0.001	0	0	—	0	0	—
Somnolence	0	0	—	0	0	—	1	0	0.315
Fatigue	0	0	—	0	0	—	0	0	—
Anorexia	2	0	0.156	0	0	—	0	2	0.153
Weight gain	0	0	—	0	0	—	0	0	—
Orthostatic	0	0	—	0	0	—	0	0	—
Hypotension	0	0	—	0	0	—	0	0	—
Agitation	0	1	0.317	0	0	—	0	0	—

Note: 4 studies did not provide the number of each specific adverse event, so they are not included in this table.

**Table 4:** Summary of comparisons of 1, 2, 4, and 6-week HAMD reduction among the patients receiving combination of Shuganjieyu capsule and regular antidepressant versus regular antidepressants.

Outcome or subgroup	Studies	Number of patients	Heterogeneity (*p*/*I*^2^)	Subgroup difference (*p*/*I*^2^)	Mean difference	*P*
8-week HAMD reduction	1	100	Not applicable	Not applicable	3.2 (1.34, 5.06)	0.0007
vs. paroxetine	1	100	Not applicable	—	3.2 (1.34, 5.06)	0.0007
6-week HAMD reduction	3	236	0.38/0%	0.92/0%	4.00 (2.72, 5.28)	<0.00001
Vs. citalopram	2	176	0.16/48%	—	4.04 (2.54, 5.54)	<0.00001
Vs. paroxetine	1	60	Not applicable	—	3.89 (1.44, 6.34)	0.002
4-week HAMD reduction	2	156	0.40/0%	0.40/0%	3.33 (1.94, 4.73)	<0.00001
Vs. citalopram	1	56	Not applicable	—	4.00 (1.90, 6.10)	0.0002
Vs. paroxetine	1	100	Not applicable	—	2.80 (0.92, 4.68)	0.003
2-week HAMD reduction	2	156	0.31/2%	0.31/2.4%	2.69 (1.34, 4.03)	<0.0001
Vs. citalopram	1	56	Not applicable	—	2.00 (0.11, 3.89)	0.04
Vs. paroxetine	1	100	Not applicable	—	3.40 (1.48, 5.32)	0.0005
1-week HAMD reduction	2	116	0.66/0%	0.66/0%	2.27 (0.69, 3.86)	0.005
Vs. citalopram	1	56	Not applicable	—	2.00 (0.01, 3.99)	0.05
Vs. paroxetine	1	60	Not applicable	—	2.75 (0.12, 5.38)	0.04

The article "Efficacy and Safety of Shuganjieyu Capsule Alone or in Combination with Other Antidepressants in the Treatment of Postpartum Depression: A Meta-Analysis" was published in 2022. Journal: Evid Based Complement Alternat Med.

**Table 5:** Summary and comparison of each adverse event among the patients receiving combination of Shuganjieyu capsule and regular antidepressant versus regular antidepressants.

Intervention	Shuganjieyu plus citalopram vs. citalopram in 3 studies [45–47]			Shuganjieyu plus sertraline vs. sertraline in 1 study [48]		
Study	Experiment (*n* = 148)	Control (*n* = 148)	*P*	Experiment (*n* = 32)	Control (*n* = 32)	*P*
Flatulence	0	0	—	3	0	0.076
Dry mouth	6	4	0.52	0	0	—
Headache	4	3	0.702	0	0	—
Dizziness	1	0	0.316	0	0	—
Insomnia	0	0	—	0	0	—
Constipation	0	0	—	0	0	—
Hand tremor	0	0	—	0	0	—
Nausea/vomiting	8	7	0.792	2	2	1
Blurred vision	0	1	0.316	0	0	—
Tachycardia	0	0	—	0	0	—
Somnolence	7	7	1	3	4	0.689
Fatigue	1	1	1	0	0	—
Anorexia	0	0	—	0	0	—
Weight gain	0	0	—	0	0	—
Orthostatic	0	0	—	0	0	—
Hypotension	0	0	—	0	0	—
Agitation	0	0	—	0	0	—

## Data Availability

The data generated or analyzed during this study are included within the article.
